The article "Long intergenic non-protein-coding RNA 467 promotes tumor progression and angiogenesis via the microRNA-128-3p/vascular endothelial growth factor C axis in colorectal cancer" was retracted in 2026. Reasons: concerns about the data; concerns about the results or conclusions.

# Long intergenic non-protein-coding RNA 467 promotes tumor progression and angiogenesis via the microRNA-128-3p/vascular endothelial growth factor C axis in colorectal cancer

**DOI:** 10.1080/21655979.2022.2074666

**Published:** 2022-05-19

**Authors:** Lisha Chang, Peipei Yang, Chun Zhang, Jing Zhu, Yirao Zhang, Yang Wang, Jie Ding, Keming Wang

**Affiliations:** a Department of Oncology, Second Affiliated Hospital, Nanjing Medical University, Nanjing, Jiangsu, China; b Department of Oncology, Nanjing First Hospital, Nanjing Medical University, Nanjing, Jiangsu, China

**Keywords:** Colorectal cancer, LINC00467, miR-128-3p, angiogenesis, VEGFC

## Abstract

Long non-coding RNAs (lncRNAs) are important regulators and biomarkers of tumorigenesis and tumor metastasis. Long intergenic non-protein-coding RNA 467 (LINC00467) is associated with various cancers. However, the role and mechanism of LINC00467 in colorectal cancer (CRC) promotion are poorly understood. This study aimed to present new details of LINC00467 in the progression of CRC. Reverse transcription–polymerase chain reaction demonstrated that the expression level of LINC00467 in CRC tissues and cell lines was significantly upregulated, which was closely related to the clinical features of CRC. Cell and animal studies showed that the downregulation of LINC00467 expression in CRC cells significantly inhibited cell proliferation, metastasis, and angiogenesis. Moreover, the overexpression of LINC00467 accelerated CRC promotion. Bioinformatics analysis and luciferase reporter assay confirmed that LINC00467 binds to miR-128-3p. Rescue experiments manifested that decreased miR-128-3p level reversed CRC cell inhibition by silencing LINC00467. Furthermore, vascular endothelial growth factor C (VEGFC) was identified as a target of miR-128-3p that could reverse the inhibition of cell growth that is mediated by miR-128-3p. Altogether, our results showed that LINC00467 contributes to CRC progression and angiogenesis via the miR-128-3p/VEGFC axis. Our findings expand the understanding of the mechanisms underlying CRC and suggest potential targets for clinical strategies against CRC.

## Highlights

- Long non-coding RNA LINC00467 and VEGFC are elevated in CRC tissues and cells.
- YTHDC1 is closely related to LINC00467 overexpression in CRC.
- LINC00467 upregulation promotes CRC progression and angiogenesis.
- LINC00467 is a competing endogenous RNA of miR-128-3p to regulate VEGFC expression.
- LINC00467 targets the miR-128-3p/VEGFC axis to promote CRC malignant behaviour.

## Introduction

Colorectal cancer (CRC) is one of the most prevalent malignancies and is usually associated with a fatal course. CRC results from the accumulation of genetic and epigenetic changes that alter the expression of protein-coding and non-coding RNAs [1–5]. Despite improvements in diagnosis and therapy, CRC can still result in a poor prognosis, as proven by the low 5-year survival rate (<50%) and frequent metastasis [6]. The management of CRC remains a clinical challenge. Treatment failure is mainly attributed to rapid tumor cell proliferation, increased angiogenesis, and distant metastasis, although the underlying mechanisms are poorly understood [7,8]. Clarifying the molecular basis of tumor proliferation, vascularization, and metastasis is critical for the development of novel therapies that can prevent tumor recurrence and progression in CRC.

The article "Long intergenic non-protein-coding RNA 467 promotes tumor progression and angiogenesis via the microRNA-128-3p/vascular endothelial growth factor C axis in colorectal cancer" was retracted in 2026. Reasons: concerns about the data; concerns about the results or conclusions.

Less than 2% of the human genome encodes for proteins, indicating that more than 98% of the region is non-coding, called non-coding RNAs (ncRNAs) [9]. Long non-coding RNAs (lncRNAs) have some common properties, including a nucleotide length of more than 200, lack of protein-coding ability, and transcription by RNA polymerase II [9,10]. Previous studies have reported increasing evidence for the regulatory functions of lncRNAs in cell proliferation, migration, invasion, apoptosis, and drug resistance in numerous malignancies, including CRC [11–13]. In this study, we found that the expression level of LINC00467 in CRC tissues and cell lines was significantly upregulated, which was strongly associated with the short survival time of patients with CRC. However, how LINC00467 is currently involved in CRC remains unclear.

Accumulating evidence has shown that some lncRNAs function as microRNA(miRNA) sponges, thereby antagonizing their functions [14]. Furthermore, aberrant lncRNA and miRNA expression has been observed in CRC [15–17]. Interestingly, LINC00467 has recently been reported to promote the development of malignancies by adsorbing miRNA. For example, in head and neck squamous cell carcinoma, LINC00467 regulates transcription factor AP-2 alpha (TFAP2A) expression as a ceRNA by adsorbing microRNA-1285-3p, thus inducing invasive changes in the tumor and inhibiting the apoptosis of cancer cells [18]. Additionally, the development of prostate carcinoma could be promoted by LINC00467 through the microRNA-494-3p/signal transducer and activator of the transcription 3 (STAT3) axis [19]. Moreover, studies have shown that miR-128-3p acts as a tumor suppressor of various genes in CRC [20,21].

Vascular endothelial growth factor (VEGF) is the most potent pro-angiogenic factor because of its mitogenic function [22,23]. VEGFC is a member of the VEGF family, and it also induces angiogenesis via the VEGFC/VEGFR2 or VEGFC/VEGFCR3 axis [24]. Angiogenesis is a pivotal process that enables tumor invasion and metastasis [25,26]. Blood vessels transport nutrients and metabolites that accelerate tumor growth and invasion and provide transport pathways for tumor cell migration. The introduction of new blood vessels is also required for the formation and growth of metastatic lesions [27]. Increasing evidence indicates that lncRNAs play an important role in tumor angiogenesis [28,29]. However, whether LINC00467 is associated with the angiogenesis phenotype in CRC has not been reported thus far, and further investigation is necessary.

The article "Long intergenic non-protein-coding RNA 467 promotes tumor progression and angiogenesis via the microRNA-128-3p/vascular endothelial growth factor C axis in colorectal cancer" was retracted in 2026. Reasons: concerns about the data; concerns about the results or conclusions.

In this study, we hypothesized that LINC00467 plays a role in CRC by regulating miR-128-3p /VEGFC. The present study aimed to investigate the new role and mechanism of LINC00467 in CRC and provide a theoretical basis for elucidating the mechanism underlying the progression of this fatal disease.

## Materials and methods

### Clinical data

Twenty-seven pairs of CRC and adjacent non-tumor tissue samples were obtained from patients who underwent surgery at The Second Affiliated Hospital of Nanjing Medical University. None of the included patients had received radiotherapy, chemotherapy, or other preoperative treatments. CRC diagnosis was confirmed by pathological examination. Ethical approval for this study was obtained from the Medical Ethics Committee of The Second Affiliated Hospital, Nanjing Medical University (approval no. [2019]-KY-121) . All patients were fully informed, and signed consent forms were obtained. Tissue samples were processed by surgical resection and liquid nitrogen for flash freezing. The storage temperature was −80°C.

### Cell culture and transfection

The cell strains selected for this study were HT-29, HCT-116, SW480, SW620, DLD1, LOVO human CRC cells, normal intestinal epithelial fetal human colon (FHC) cells (Cell Bank of the Chinese Academy of Sciences, Shanghai, China), and human umbilical vein endothelial cells (HUVECs; American Type Culture Collection, Manassas, VA, USA). Dulbecco’s modified Eagle’s medium (DMEM; Gibco, Grand Island, NY, USA) containing 10% fetal bovine serum (FBS) and 1% penicillin/streptomycin was used. The cell culture samples were incubated at 37°C and 5% CO_2_ [30]. Next, 2 μM LINC00467-siRNA (si-LINC00467), 2 μM control-siRNA, 50 nM miR-128-3p inhibitor, 50 nM miR-128-3p mimic, 50 nM inhibitor control, and 50 nM mimic control were synthesized using RiboBio Co. (Guangzhou, China). Before use in experiments, the samples were examined to guarantee the logarithmic growth of the cells. Then the cells (at a density of 0.5 × 10^6^ cells/well) were grown in 6-well plates until they reached 70–80%; plasmid (0.4 µg), small interfering RNA (siRNA), inhibitor, and mimics (50 nM) diluted with the Opti-MEM medium (Thermo Fisher Scientific, USA) were transfected into cells using Lipofectamine 2000 (Invitrogen, Carlsbad, CA, USA) or X-tremeGENE transfection reagent (Thermo Fisher Scientific, USA); 24–48 h after transfection at 37°C, the cells were collected to determine the transfection efficiency by quantitative reverse transcription–polymerase chain reaction (qRT-PCR) [29]. Interference sites with good transfection efficiency were selected for subsequent experiments.

The article "Long intergenic non-protein-coding RNA 467 promotes tumor progression and angiogenesis via the microRNA-128-3p/vascular endothelial growth factor C axis in colorectal cancer" was retracted in 2026. Reasons: concerns about the data; concerns about the results or conclusions.

### qRT-PCR

Total RNA from tissues or cells was isolated using the TRIzol reagent (Invitrogen, Carlsbad, CA, USA). The purity and concentration of the extracted RNA were determined using a spectrophotometer, and the concentrations for each pair of samples were adjusted so that they were equivalent. We reverse transcribed 1 μg RNA into cDNA using a Qiagen kit (Qiagen, Valencia, CA, USA), and qRT-PCR was performed on StepOnePlus™ Real-Time PCR System (Applied Biosystems; Shanghai, China) using the SYBR Premix Ex Taq Kit (Takara, Otsu, Japan), according to the manufacturer’s protocol [30]. PCR cycling conditions were as follows: 95°C for 2 min, 40 cycles of 95°C for 5 s, 60°C for 34s, and 68°C for 20s. PCR was performed in a 20-µL reaction. Stem-loop qRT-PCR detected miR-128-3p expression, and the results were normalized to U6 gene expression levels. The results of LINC00467 and VEGFC were normalized to the level of glyceraldehyde 3-phosphate dehydrogenase (GAPDH) [29]. The 2^−ΔΔCt^ method was used to determine relative gene expression levels, and GAPDH was used as the internal reference gene. All primer sequences were synthesized and purchased from Invitrogen Shanghai Trading Co. Ltd. (Shanghai, China). Primer sequences are presented in Table 1.

**Table 1.** Primer sequences

Gene	Sequence (5’-3’)-F	Sequence (5’-3’)-R
LINC00467	CAGGAAGCCAGACAGATTCA	AGCCCAGTTTCAGTCCCTCT
GAPDH	GAA GGT GAA GGT CGG AGT C	GAA GAT GGT GAT GGG ATTTC
U6	CTCGCTTCGGCAGCACA	AACGCTTCACGAATTTGCGT
YTHDC1	AAGTCGGCTCATCTCACCAA	ACTGGTTCTCGACGGGATG
VEGFC	GCCACGGGAGGTGTGTATAG	ATCGGCAGGAAGTGTGATTG
miR-128-3p	TCACAGTGAACCGGTC	CAGTGCGTGTCGTGGAGT

### Cell counting kit-8 assay

Cell counting kit-8 (CCK-8) assay was used to detect the viability of transfected cells, and the method was performed according to a previous experiment [31]. Twenty-four hours after transfection, the cells in the medium were digested with 0.25% trypsin, and the cell suspension was collected and counted and then seeded into 96-well plates, with 5 wells in each group. Each well contained 2 × 10^3^ cells and 100 μL of the medium at 37°C, with 5% CO_2_ for 0, 1, 2, 3, 4, and 5 days. The final selection of a culture time of 5 days is because we found that 5 days is the time point of the maximum optical density (OD) value of the CCK-8 test and the time node most suitable for observing the OD value through the preliminary experiment. Subsequently, 10 μL of the CCK-8 solution (KeyGEN, Nanjing, China) was pipetted into individual wells of a 96-well plate. The incubation was continued for 2 h. The cell proliferation rate was measured by reading the absorbance at 450 nm using a microplate reader.

The article "Long intergenic non-protein-coding RNA 467 promotes tumor progression and angiogenesis via the microRNA-128-3p/vascular endothelial growth factor C axis in colorectal cancer" was retracted in 2026. Reasons: concerns about the data; concerns about the results or conclusions.

### 5-Ethynyl-2′-deoxyuridine incorporation assay

Tumor cell proliferative capacity was evaluated using the 5-ethynyl-2*′*-deoxyuridine (EdU) assay kit (RiboBio). Twenty-four hours after transfection, the cells were inoculated into 96-well plates at a density of 8 × 10^3^ cells per well, and after subsequent 24 h incubation, the cell samples were incubated with 50 µM EdU at 37°C for 2 h and subsequently fixed with 4% paraformaldehyde for 30 min. The fixed cells were rinsed with 2 mg/mL glycine for 5 min, and phosphate-buffered saline (PBS) with 0.5% Triton X-100 was subsequently applied for 10 min. The cells were stained with 1× Apollo staining solution for 30 min. After rinsing with PBS (0.5% Triton X-100) for 10 min, the cells were incubated in 100 mL of 1× Hoechst 33,342 for 30 min. Subsequently, the cells were fixed in 4% paraformaldehyde and stained with DAPI. Finally, cell counting was performed using fluorescence microscopy to quantify the percentage of EdU-positive cells [32].

### Cell invasion and migration assay

Tumor cells’ migratory and invasive abilities were evaluated using the Transwell assay. Twenty-four hours after transfection, the cells in the medium were digested with 0.25% trypsin; by cell counting, transfected CRC cells were seeded into a 24-well plate containing a Transwell chamber with 6 × 104 cells/well concentration. A total of 200 μL of the serum-free medium was added to the upper chamber, and cells were seeded, whereas 800 μL of DMEM with 15% FBS was added to the lower chamber. After incubation in a cell incubator at 37°C with 5% CO_2_ for 24–48 h, the inserted membrane was fixed using methanol and stained with 0.1% crystal violet. The upper surface of the membrane was swabbed, and the migrated cells on the lower surface were photographed using an inverted research microscope [30]. For the cell invasion assay, a layer of Matrigel gel was applied to the upper side of the membrane, and the rest was consistent with the cell migration assay.

### Colony formation assay

Colony formation assay was performed to evaluate the cells’ colony formation ability. Cells were counted 24 h after transfection, and the cells (300–500 cells/well) were seeded in 6-well plates with 2 mL of medium containing 10% FBS per well and cultured at 37°C with 5% CO_2_ for 14 days. The medium was replaced every 5 days. After 14 days, the medium was discarded, and the cells were washed with PBS twice and fixed with methanol. The cells were stained with 0.1% crystal violet and incubated at room temperature for 30 min. Photographs were taken for colony count [33].

The article "Long intergenic non-protein-coding RNA 467 promotes tumor progression and angiogenesis via the microRNA-128-3p/vascular endothelial growth factor C axis in colorectal cancer" was retracted in 2026. Reasons: concerns about the data; concerns about the results or conclusions.

### Matrigel tube formation assay

This assay was used to evaluate the angiogenic ability of the HUVECs in vitro. Matrigel was thawed at 4°C for 10 h, and the 96-well plates were placed in advance at 4°C for cooling. Then, 60 µL of Matrigel was evenly spread onto the bottom of a 96-well plate for each well, and the ice was shaken horizontally. The plate was incubated for 30 min at 37°C, and the Matrigel solidified during this period. HUVECs grown to 80% confluence were washed twice with PBS and digested with 0.25% trypsin. Then, the supernatant of CRC cells collected 24 h after transfection was used to resuspend HUVECs and counted, the 200 μl cell suspension (2 × 10^4^ cells/well) was transferred to Matrigel-coated wells [34]. After incubation at 37°C with 5% CO_2_ for 16–18 h, the formed tubes were detected with inverted microscopy at low magnification, and photos were recorded. The number of meshes and branches was determined using ImageJ software (National Institutes of Health, Bethesda, MD, USA).

### Subcellular RNA fractionation

The NE-PER Nuclear and Cytoplasmic Extraction Kit (Thermo Fisher Scientific, Waltham, MA, USA) was used to extract nuclear and cytosolic RNA, according to the manufacturer’s instructions. Briefly, 10 × 10^4^ target cells were suspended in 300 μl cell fractionation buffer and centrifuged at 500 × g at 4°C for 5 min. The cytoplasmic portion was isolated and placed in fresh RNase-free test tubes. The nuclear pellet was then cleaved using a cell disruption buffer. We added the same volume of 2X lysis/binding solution as the RNA lysate to the nuclear lysates and cytoplasmic fractions before treatment with 100% ethanol. The sample mixture was then separated by RNA separation. qRT-PCR was used to detect nuclear and cytosolic RNA levels with U6 and β-actin, respectively. GAPDH was used as the cytoplasmic reference, and U6 was used as the nuclear reference [35,36].

### Luciferase reporter assay

To detect the binding between miR-128-3p and LINC00467/VEGFC, the cells in the logarithmic growth phase were counted and digested with 0.25% trypsin to produce a cell suspension. The cell suspension (approximately 2 × 10^4^ cells) was seeded in 24-well culture plates at 37°C in a 5% CO_2_ incubator until the degree of cell fusion reached approximately 60%. Subsequently, HEK293 subcultures were co-transfected with miR-128-3p mimic or negative control miRNA and wild-type (WT)-LINC00467/mutant (MUT)-LINC00467 or WT-VEGFC/MUT-VEGFC. Forty-eight hours after transfection, the fluorescent reporter protein was detected. Finally, the dual-luciferase reporter assay (Promega, Madison, WI, USA) was used to evaluate luciferase activity by measuring the absorbance on a microplate reader, according to the manufacturer’s instructions [36].

The article "Long intergenic non-protein-coding RNA 467 promotes tumor progression and angiogenesis via the microRNA-128-3p/vascular endothelial growth factor C axis in colorectal cancer" was retracted in 2026. Reasons: concerns about the data; concerns about the results or conclusions.

### Zebrafish xenograft model

LOVO cells transfected with siRNA for 24 h were collected and washed with HBSS three times. Then added 1 μl CM-DiI (Invitrogen, USA) stain at 37°C for 5 min, followed by 15 min at 4°C, then washed with HBSS three times. Forty-eight hours post-fertilization (hpf), embryos of type AB wild zebrafish were fixed on a low melting point agarose gel. The LoVo cells were injected into the perivitelline space (PVS) with 400 cells/embryos. The xenografts injected with LoVo cells were cultured in a 34°C incubator and observed under a microscope on the second day after the tumor cells were transplanted. Zebrafish embryos successfully transplanted with relatively similar sizes were selected and cultured at 34°C until the end of the experiment. The juveniles at 4 day post-injection(dpi) were fixed with low melting gel for microscopic imaging [37].

### Statistical analysis

Each result is expressed as the mean ± standard deviation of three independent experiments. SPSS v17.0 software (SPSS Inc., Chicago, IL, USA) and Prism v7 software (GraphPad, La Jolla, CA, USA) were used for conducting the statistical calculations. A one-way analysis of variance was used to compare multiple groups. The difference between the two groups was evaluated using Student’s t-test. Differences were considered statistically significant at P < 0.05.

## Results

In this study, we investigated the role of LINC00467 and its downstream molecular mechanisms in CRC. Our data showed that LINC00467 expression was upregulated in CRC, and silencing of LINC00467 inhibited the proliferation, migration, invasion, and angiogenesis of CRC cells. Based on findings of bioinformatics analysis and a series of cell-functional assays, we identified that LINC00467 plays a role in CRC by regulating miR-128-3p/VEGFC. Our findings enrich the understanding of the mechanisms underlying CRC progression and may serve as molecular markers for CRC treatment.

### LINC00467 is upregulated in CRC tissue and cells

To identify lncRNAs closely related to CRC, we downloaded publicly available datasets from The Cancer Genome Atlas (TCGA) and Gene Expression Omnibus (GEO) for bioinformatics analysis. We found that CRC tissues overexpressed LINC00467 compared to normal tissues in the GSE21510 dataset (Figure 1(a, b)). An analysis of common CRC datasets in the Gene Expression Profiling Interactive Analysis database (http://gepia.cancer-pku.cn/) revealed significantly increased LINC00467 levels in colorectal adenocarcinoma samples (Figure 1(c)). Additionally, TCGA analysis (http://tumorsurvival.org/index.html) showed that a higher pathologic stage of CRC was associated with higher LINC00467 expression (Figure 1(d)). We also analyzed LINC00467 expression levels in seven CRC cell lines and FHC cells. According to qRT-PCR data, LINC00467 expression was upregulated in CRC cells compared to that in normal cells (Figure 1(e)), which is consistent with the results obtained from TCGA data analysis. Therefore, according to the expression of LINC00467 in CRC cell lines, SW620 and LOVO cell lines with higher expression levels were selected for the knockdown, while SW480 cell lines with the lowest high expression levels were overexpressed in subsequent experiments. We also analyzed LINC00467 expression in tumors and adjacent normal tissues surgically resected from patients with CRC at our hospital. LINC00467 expression was upregulated in tumor tissue samples (figure 1(f)) and was associated with shorter recurrence-free and overall survival rates (Figure 1(g, h)). These results suggested that LINC00467 overexpression is involved in CRC progression.

The article "Long intergenic non-protein-coding RNA 467 promotes tumor progression and angiogenesis via the microRNA-128-3p/vascular endothelial growth factor C axis in colorectal cancer" was retracted in 2026. Reasons: concerns about the data; concerns about the results or conclusions.

**Figure 1.** LINC00467 expression in colorectal cancer (CRC). a, b Depending on Gene Expression Omnibus (GEO) (GEO: GSE21510) and The Cancer Genome Atlas (TCGA) datasets, relative LINC00467 expression in CRC tissues was compared with that in non-tumor tissues. c Depending on the findings of the Gene Expression Profiling Interactive Analysis database (GEPIA) database, LINC00467 expression in CRC was assessed (colon adenocarcinoma, COAD; rectal adenocarcinoma, READ). d Depending on the information in the TCGA database, the relevance of LINC00467 expression with CRC pathologic stages was assessed. e Analysis of LINC00467 expression levels in CRC cell lines by reverse transcription–polymerase chain reaction. f Relative LINC00467 expression in CRC tissues was assessed by comparing it with that in non-tumor samples (n = 27). g, h Depending on the information in the GEPIA and A comprehensive resource for lncRNAs from Cancer Arrays (InCAR) databases, the clinical impacts of abnormal LINC00467 expression levels on the CRC disease-free survival (DFS) and overall survival (OS) were assessed. Data are presented as mean ± standard deviation (SD); *P < 0.05, **P < 0.01, ***P < 0.001, ****P < 0.0001.

### YTHDC1 may be associated with the expression of LINC00467 in CRC

LINC00467 is located at 1q32.3 and has six exons (Figure 2(a)). The secondary structure is shown in Figure 2(b). The low coding potential of LINC00467 was predicted using the LNCipedia (https://lncipedia.org/) (Figure 2(c)). Genes functionally related to LINC00467 were analyzed using co-expression network (Figure 2(d)). Then, the following criteria were used to screen the target gene: (1) positively correlated with LINC00467, and the correlation was greater than 0.2; (2) it had been reported to be highly expressed in CRC; (3) it had been reported to have a function in CRC; (4) it has been reported to be co-expressed with lncRNAs. Finally, we chose YTH domain-containing 1 (YTHDC1) as the target gene. Subsequently, we identified putative YTHDC1-binding sites in LINC00467 using annonlnc (http://annolnc.gao-lab.org/index.php) (Figure 2(e)). We analyzed the starBase database from the TCGA data portal (https://starbase.sysu.edu.cn/) and found a positive association between YTHDC1 and LINC00467 levels in CRC (figure 2(f, g)). We constructed an RNA interference plasmid targeting YTHDC1 and evaluated its knockdown efficiency by qRT-PCR (Figure 2(h)). This construct effectively reduced LINC00467 expression in LOVO and SW620 cells (Figure 2(i)). These data demonstrate that YTHDC1 may be associated with the expression of LINC00467 in CRC.

The article "Long intergenic non-protein-coding RNA 467 promotes tumor progression and angiogenesis via the microRNA-128-3p/vascular endothelial growth factor C axis in colorectal cancer" was retracted in 2026. Reasons: concerns about the data; concerns about the results or conclusions.

**Figure 2.** YTHDC1 may be associated with the expression of LINC00467 in CRC. a Position of LINC00467 on the chromosome. b The AnnoLnc2 database was used to obtain the secondary structure of LINC00467. c The LNCipedia database was used to predict the coding capability of LINC00467. d Bioinformatics prediction of RNA binding protein (RBP). e The AnnoLnc2 database was used to display the binding site of YTHDC1 and LINC00467. f, g The Starbase database was used to analyze the correlation between YTHDC1 and LINC00467. h In LOVO and SW620 cells, the interference efficiency of YTHDC1 was assessed using reverse transcription–polymerase chain reaction (qRT-PCR). i LINC00467 expression was determined by the qRT-PCR assay subsequent to YTHDC1 knockdown by transfection. Data are presented as mean ± standard deviation (SD); *P < 0.05, **P < 0.01, ***P < 0.001, ****P < 0.0001.

### LINC00467 promotes CRC cell proliferation

To analyze the phenotypic effect of LINC00467 on CRC, we utilized the Kyoto Encyclopedia of Genes and Genomes. It was confirmed that LINC00467 had close relevance with the occurrence and progression of CRC (Figure 3(a)). To determine the biological role of LINC00467, we measured LINC00467 expression levels in LINC00467-depleted LOVO and SW620 cells, as well as in SW480 cells exogenously overexpressing LINC00467 (Figure 3(b, c)). LINC00467 knockdown inhibited CRC cell proliferation and colony-forming ability (Figure 3(d, f)), whereas LINC00467 overexpression had a contrasting effect (Figure 3(e, g)). The EdU assay confirmed that LINC00467 knockdown and overexpression significantly suppressed and enhanced the proliferative capacity of CRC cells, respectively (Figure 3(h, i)).

The article "Long intergenic non-protein-coding RNA 467 promotes tumor progression and angiogenesis via the microRNA-128-3p/vascular endothelial growth factor C axis in colorectal cancer" was retracted in 2026. Reasons: concerns about the data; concerns about the results or conclusions.

**Figure 3.** LINC00467 promotes colorectal cancer (CRC) cell proliferation in vitro. a Kyoto Encyclopedia of Genes and Genomes pathway analysis. b, c In CRC cell samples, the interference and overexpression efficiency of LINC00467 were verified by reverse transcription–polymerase chain reaction (qRT-PCR). d For LINC00467 knockdown, the Cell Counting Kit (CCK)-8 assay assessed CRC cell viability. e For LINC00467 overexpression, the CCK-8 assay assessed CRC cell viability. f For LINC00467 knockdown, colony-forming assays assessed CRC cell proliferation. g For LINC00467 overexpression, colony-forming assays assessed CRC cell proliferation. h For LINC00467 knockdown, EdU assays assessed CRC cell proliferation. i For LINC00467 overexpression, EdU assays assessed CRC cell proliferations. Data are presented as mean ± standard deviation (SD); *P < 0.05, **P < 0.01, ***P < 0.001, ****P < 0.0001.

### LINC00467 promotes CRC cell migration and invasion as well as vascular endothelial cell angiogenesis

We further investigated the involvement of LINC00467 in the aggressive behavior of CRC cells. According to the Transwell Matrigel assay, LINC00467 silencing contributed to a marked decrease in the migration and invasion of CRC cells (Figure 4(a, b)). By contrast, LINC00467 overexpression enhanced the migration and invasion of CRC cells (Figure 4(c)). Given the importance of angiogenesis in tumor development, we used the transfected CRC cell supernatant and resuspended HUVECs to observe the angiogenesis of HUVECs and found that the tube-forming ability of these cells was decreased in the presence of the supernatant collected from LINC00467-depleted cells (Figure 4(d)), whereas a contrary effect was observed in the supernatant collected from LINC00467-overexpressing cells (Figure 4(e)). These findings suggest that elevated LINC00467 expression enhances CRC cell proliferation, metastasis, and angiogenesis.

**Figure 4.** LINC00467 promotes colorectal cancer (CRC) cell migration, invasion, and angiogenesis of human umbilical vein endothelial cells (HUVECs) in vitro. a, b Transwell assays examined LOVO and SW620 cells transfected with LINC00467 siRNAs. c Transwell assays examined SW480 cells transfected with pcDNA-LINC00467. d, e Angiogenesis assay described the angiogenesis of HUVECs (number of branches, meshes), which co-cultured with CRC cells transfected with LINC00467 siRNAs or pcDNA-LINC00467. Data are presented as mean ± standard deviation (SD); *P < 0.05, **P < 0.01, ***P < 0.001, ****P < 0.0001.

The article "Long intergenic non-protein-coding RNA 467 promotes tumor progression and angiogenesis via the microRNA-128-3p/vascular endothelial growth factor C axis in colorectal cancer" was retracted in 2026. Reasons: concerns about the data; concerns about the results or conclusions.

### LINC00467 is a ceRNA for miR-128-3p

To elucidate how LINC00467 participates in CRC progression, we performed bioinformatics analysis to predict the subcellular distribution of LINC00467 in various cells and observed predominantly cytosolic LINC00467 localization (Figure 5(a)). Subcellular fractionation of CRC cells confirmed that LINC00467 was more abundant in the cytoplasm than in the nucleus of LOVO, SW620, and SW480 cells (Figure 5(b)). As ceRNAs, lncRNAs control target gene expression by sponging miRNAs, implying that LINC00467 can act as a ceRNA in CRC [38–41]. To investigate whether LINC00467 has this function, we predicted miRNAs that target LINC00467 by searching miRDB (www.mirdb.org/custom.html), DIANA (carolina.imis.athena-innovation.gr/diana_tools/web/index.php?r = site%2 Findex), and Jefferson (https://cm.jefferson.edu/). Among the findings, miR-299-5p, miR-216a-3p, and miR-128-3p shared a highly conserved sequence with LINC00467 (Figure 5(c)), but only miR-128-3p showed a negative correlation with LINC00467 (Figure 5(d)). This finding was consistent with the predicted results (Figure 5(e)). Therefore, we selected miR-128-3p for subsequent analysis. Bioinformatics analysis was performed to identify putative miR-128-3p-binding sites in the 3′-untranslated region (UTR) of LINC00467 (figure 5(f)). Based on the predicted results, the WT and MUT LINC00467 plasmids were constructed for the luciferase reporter assay. The miR-128-3p mimic markedly inhibited the luciferase activity of LINC00467-3′-UTR-WT but showed no obvious effect on that of LINC00467-3′-UTR-MUT (Figure 5(g)). In conclusion, LINC00467 acts as a miR-128-3p sponge.

**Figure 5.** LINC00467 is a ceRNA against miR-128-3p. a Bioinformatics analyses predicted the subcellular distribution of LINC00467 in various cells. b Subcellular localization of LINC00467 in colorectal cancer (CRC). The nuclear marker was U6, and the cytosol marker was glyceraldehyde 3-phosphate dehydrogenase (GAPDH). c Venn diagram showing the overlap between predicted LINC00467 targets, depending on miRDB, DIANA, and Jefferson databases. d Reverse transcription–polymerase chain reaction (qRT-PCR) assays show changes in miR-299-5p, miR-216a-3p, and miR-128-3p expression levels after transfection with LINC00467 siRNAs or pcDNA-LINC00467. e Depending on the information in the Starbase database, the correlation between miR-128-3p and LINC00467. f Putative binding site between LINC00467 and miR-128-3p identified from DIANA online software. g Luciferase reporter assay assessed the interaction between LINC00467 and miR-128-3p. Data are presented as mean ± standard deviation (SD); *P < 0.05, **P < 0.01, ***P < 0.001, ****P < 0.0001.

The article "Long intergenic non-protein-coding RNA 467 promotes tumor progression and angiogenesis via the microRNA-128-3p/vascular endothelial growth factor C axis in colorectal cancer" was retracted in 2026. Reasons: concerns about the data; concerns about the results or conclusions.

### LINC00467 interacts with miR-128-3p to enhance CRC proliferation, metastasis, and angiogenesis

These results indicated that LINC00467 targets miR-128-3p. To determine whether LINC00467 contributes to the malignant progression of CRC through miR-128-3p, we designed an inhibitor of miR-128-3p (Figure 6(a)) that was transfected into LINC00467-depleted CRC cells. According to the CCK-8 and colony formation assays, while LINC00467 silencing decreased the proliferative and colony-forming abilities of CRC cells, the inhibitory effects could be reversed by the miR-128-3p inhibitor (Figure 6(b, c)). LINC00467 depletion also suppressed CRC cell migration and invasion, which were restored by the miR-128-3p inhibitor (Figure 6(d, e)). The proangiogenic effect of the CRC cell supernatant was assessed in HUVECs. Angiogenesis was reduced in HUVECs treated with the supernatant from LINC00467 knockdown cells compared to that from control cells. Inhibition of both LINC00467 and miR-128-3p promoted angiogenesis in HUVECs compared to that in the LINC00467 knockdown + negative control miRNA group (figure 6(f)). Accordingly, the involvement of LINC00467 in CRC development relies on miR-128-3p regulation.

**Figure 6.** LINC00467 enhances colorectal cancer (CRC) progression by sponging miR-128-3p. a Reverse transcription–polymerase chain reaction (qRT-PCR) measured miR-128-3p interference efficiency in CRC cells. In LOVO and SW620 cells, functional rescue experiments including the CCK-8 assay were conducted. b, Colony-forming assays c, Transwell assays d, e and angiogenesis assay f. Data are presented as mean ± standard deviation (SD); *P < 0.05, **P < 0.01, ***P < 0.001, ****P < 0.0001.

### VEGFC/miR-128-3p axis regulates malignant cell behaviors in CRC

Bioinformatics analysis revealed a putative miR-128-3p-binding site in the 3′-UTR of the VEGFC gene (Figure 7(a)). We also found that miR-128-3p expression was negatively associated with VEGFC expression (Figure 7(b)). In luciferase reporter assays, co-transfection of VEGFC 3′-UTR-WT and VEGFC 3′-UTR-MUT plasmids with either the miR-128-3p mimic or negative control into CRC cells was conducted. Consequently, the luciferase activity of VEGFC 3′-UTR-WT was suppressed by inhibition of the miR-128-3p mimic (Figure 7(c)), suggesting that VEGFC is a potential target for miR-128-3p. qRT-PCR analysis verified that VEGFC expression was upregulated in CRC specimens (Figure 7(d)), and high VEGFC expression was significantly associated with the prognosis of CRC patients (Figure 7(e)). To assess whether both miR-128-3p and LINC00467 could alter VEGFC expression in CRC, we evaluated VEGFC expression levels in LOVO and SW620 cells expressing the miR-128-3p-mimic and LINC00467 siRNA. Quantitative analysis revealed that both miR-128-3p and LINC00467 modulated VEGFC expression. Overexpression of miR-128-3p and knockdown of LINC00467 significantly decreased VEGFC expression in CRC cells (figure 7(f, g)).

The article "Long intergenic non-protein-coding RNA 467 promotes tumor progression and angiogenesis via the microRNA-128-3p/vascular endothelial growth factor C axis in colorectal cancer" was retracted in 2026. Reasons: concerns about the data; concerns about the results or conclusions.

**Figure 7.** Vascular endothelial growth factor C (VEGFC) is a direct target of miR-128-3p and upregulated VEGFC expression counteracts the functions of miR-128-3p on colorectal cancer (CRC) cells. a Starbase online software identified putative binding sites between VEGFC and miR-128-3p. b Depending on information in the Starbase database, the correlation between miR-128-3p and VEGFC was assessed. c Luciferase reporter assay assessed the interaction between miR-128-3p and VEGFC. d Relative expression of VEGFC in CRC tissues compared with the corresponding adjacent normal tissues (n = 27). e Depending on the information in the GEPIA database, the clinical impacts of abnormal VEGFC levels on the CRC disease-free survival (DFS) and overall survival (OS) were clarified. f, g In LOVO and SW620 cells, reverse transcription–polymerase chain reaction (qRT-PCR) assessed miR-128-3p-mimic and LINC00467 SiRNAs in suppressed VEGFC expression. h The overexpression efficiency of VEGFC was verified in CRC cells by qRT-PCR. In LOVO and SW620 cells, functional rescue experiments including colony-forming assays were conducted. i, Transwell assays j, k and angiogenesis assay l. Data are presented as mean ± standard deviation (SD); *P < 0.05, **P < 0.01, ***P < 0.001, ****P < 0.0001.

To assess the miR-128-3p-mediated involvement of VEGFC in CRC cell proliferation, metastasis, and angiogenesis, VEGFC overexpression in LOVO and SW620 cells induced by pCDNA3.1-VEGFC, which could abrogate the inhibition of malignant behaviors caused by upregulated miR-128-3p expression, was confirmed with qRT-PCR (Figure 7(h)). The results of the cell proliferation (Figure 7(i)), migration, invasion (Figure 7(j, k)), and tube formation (Figure 7(l)) assays proved that the inhibitory effects on CRC cells induced by the miR-128-3p-mimic could be alleviated by VEGFC overexpression. In conclusion, the LINC00467/miR-128-3p/VEGFC axis regulates the malignant behavior of CRC cells.

### LINC00467 promotes CRC cell proliferation and migration in vivo

To further determine the effect of LINC00467 on tumor in vivo. We transplanted LoVo cells transfected with siRNA and siNC into zebrafish embryos. At 4 dpi, the yolk and trunk of the juvenile samples were photographed. We quantified this region with CM-DiI positive signals, which represented the tumor region of the yolk and trunk (Figure 8(a, c)). Compared with the siNC group, we observed that after knocking down LINC00467 in LOVO cells, the CM-DiI-positive areas in the yolk and stem were significantly smaller (Figure 8(b, d)), indicating that the proliferation (in yolk) and migration (in trunk) of LOVO cells after knockdown LINC00467 were weakened. These results are consistent with data from in vitro.

The article "Long intergenic non-protein-coding RNA 467 promotes tumor progression and angiogenesis via the microRNA-128-3p/vascular endothelial growth factor C axis in colorectal cancer" was retracted in 2026. Reasons: concerns about the data; concerns about the results or conclusions.

**Figure 8.** LINC00467 promotes CRC cell proliferation and migration in vivo. a, c LoVo cells transfected with si-LINC00467 siRNA or NC were injected into the PVS of zebrafish larvae. Images were taken using a stereomicroscope at 4 dpi. CM-DiI-positive areas in the yolk were quantified for proliferation (a), and CM-DiI-positive areas in trunk were quantified for migration (c). The regions enclosed by the black dashed curve in the segmented images were selected for calculating tumor areas in the yolk or trunk. b, d Statistical analysis of proliferation (b) and invasion (d) when knocking down LINC00467 in LOVO cells; *P < 0.05, **P < 0.01, ***P < 0.001, ****P < 0.0001.

## Discussion

Because of the lack of effective methods for early diagnosis of CRC, its survival rate is not optimistic. Therefore, research on the incidence and mechanism of CRC has become a hotspot in recent years. Increasing evidence suggests that lncRNAs and miRNAs regulate malignant phenotypes of tumors and serve as diagnostic and prognostic biomarkers [42]. For example, LINC00638 promotes immune escape in hepatocellular carcinoma by sponging microRNA-4732-3p and targeting UL16-binding protein 1 (ULBP1) [43], and the lncRNA Down syndrome critical region 8 (DSCR8) interacts with microRNA-137 to facilitate gastric cancer progression [44]. The results of this study showed that LINC00467 was significantly elevated in CRC, and LINC00467 played a tumor-promoting role in CRC by regulating miR-128-3p/VEGFC.

Some recent studies have reported the effects of LINC00467 in human malignancies. For instance, LINC00467 was highly expressed in gastric cancer and drove the malignant progression of gastric cancer through the miR-27b-3p/STAT3 axis [45]. LINC00467 was overexpressed in NSCLC, and knockdown of LINC00467 upregulated miR-125a-3p to decrease cisplatin (DDP) resistance in NSCLC cells via inhibiting SIRT6 and inactivating the ERK1/2 signaling pathway [46]. Furthermore, it was observed that LINC00467 is highly expressed in bladder cancer and can promote bladder cancer progression by regulating the NF-κB signaling pathway [47]. According to our findings, LINC00467 expression is upregulated in CRC, which could lead to tumor progression and poor prognosis in patients with CRC. LINC00467 knockdown suppresses CRC cell proliferation, metastasis and angiogenesis. Moreover, transplanted tumor growth and metastasis in zebrafish were effectively slowed by LINC00467 knockdown. These data suggested that LINC00467 is an oncogenic lncRNA in CRC. Previous studies have elucidated that LINC00467 promoted CRC proliferation and metastasis via microRNA-451a or ATP synthase–associated peptide (ASAP) [48,49]. Compared with this report, we further comprehensively examined the effects of LINC00467 on CRC proliferation, migration, invasion and angiogenesis. Excessive angiogenesis is a basic feature of cancer that contributes to tumor growth, metastasis, chemoresistance, and vascular permeability changes [50–52]. Although several lncRNAs associated with angiogenesis have been identified in CRC [53,54], few anti-angiogenic treatments are known to be effective in CRC. This study is also the first to demonstrate that LINC00467 regulates angiogenesis in CRC. Furthermore, a novel competing endogenous RNA (ceRNA) regulatory mechanism of LINC00467 in CRC was investigated in detail.

The article "Long intergenic non-protein-coding RNA 467 promotes tumor progression and angiogenesis via the microRNA-128-3p/vascular endothelial growth factor C axis in colorectal cancer" was retracted in 2026. Reasons: concerns about the data; concerns about the results or conclusions.

LncRNAs in the cytoplasm can act as natural miRNA sponges to inhibit miRNA functions and regulate mRNA expression [55]. According to the subcellular RNA fractionation assay, LINC00467 was mainly located in the cytoplasm. Subsequent experiments confirmed that miR-128-3p was a direct target of LINC00467. miR-128-3p acts as a tumor suppressor miRNA in various tumors [21,56]. More importantly, miR-128-3p was previously found to be downregulated in CRC. Functionally, overexpression of miR-128-3p inhibited CRC proliferation and metastasis [21]. We observed a negative correlation between miR-128-3p and LINC00467 expression in CRC. Moreover, the inhibitory effect of LINC00467 knockdown on the malignant behavior of cells was impaired due to decreased miR-128-3p expression. That is, LINC00467 could exert a tumor-promoting effect in CRC by sponging miR-128-3p. Furthermore, the downstream targets of miR-128-3p and its association with LINC00467 were not reported.

VEGFC is the main regulator of angiogenesis and accelerates tumor progression by promoting angiogenesis by binding to the kinase insert domain receptor (VEGFR-2) [57,58]. Increased VEGFC expression was observed in patients with CRC, and high VEGFC expression was significantly associated with the prognosis of CRC patients. Interestingly, VEGFC was shown as a downstream target of miR-128-3p. More importantly, LINC00467 can act as a sponge for miR-128-3p to promote the expression of VEGFC. Also, the anticancer activity induced by LINC00467 knockdown was significantly abolished due to the recovery of VEGFC expression. We deduced from the above data that LINC00467 promoted CRC progression and angiogenesis by regulating miR-128-3p /VEGFC. Other downstream effectors of LINC00467 may also be involved in the regulation of CRC cell malignant phenotypes, which requires further study.

The article "Long intergenic non-protein-coding RNA 467 promotes tumor progression and angiogenesis via the microRNA-128-3p/vascular endothelial growth factor C axis in colorectal cancer" was retracted in 2026. Reasons: concerns about the data; concerns about the results or conclusions.

The current study showed that YTHDC1 mainly acts as an N6-methyladenosine (m6A) reader in CRC, and YTHDC1 recognizes m6A-modified mRNAs and regulates downstream gene expression [59]. In eukaryotes, N6-methyladenosine (m6A) is the most common RNA modification and has been implicated in various steps of RNA turnover, including RNA processing, nuclear export, translational control, and RNA degradation [60]. Our study is the first to demonstrate that YTHDC1 is closely related to LINC00467 expression in CRC, suggesting that LINC00467 is regulated by a novel epigenetic mechanism, m6A. This may be used as a potential therapeutic target for CRC treatment. However, the underlying mechanism requires further research, especially at the molecular level.

## Conclusion

Overall, we found that LINC00467 expression is upregulated in CRC and is associated with poor prognosis in patients with CRC. In addition, YTHDC1 may be associated with the expression of LINC00467 in CRC. LINC00467 promoted CRC cell proliferation, migration, invasion, and angiogenesis by regulating the miR-128-3p/VEGFC axis. These findings provide a new explanation for CRC progression and expand the understanding of the mechanisms underlying CRC, suggesting potential targets for clinical treatment strategies against CRC.

## Data Availability

The data are available from the corresponding author upon reasonable request.
